# The Association between Hypertension and Depression and Anxiety Disorders: Results from a Nationally-Representative Sample of South African Adults

**DOI:** 10.1371/journal.pone.0005552

**Published:** 2009-05-14

**Authors:** Anna Grimsrud, Dan J. Stein, Soraya Seedat, David Williams, Landon Myer

**Affiliations:** 1 School of Public Health & Family Medicine, University of Cape Town, Cape Town, South Africa; 2 Department of Psychiatry & Mental Health, University of Cape Town, Cape Town, South Africa; 3 Department of Psychiatry, University of Stellenbosch, Stellenbosch, South Africa; 4 Department of Society, Human Development and Health, Harvard School of Public Health, Boston, Massachusetts, United States of America; London School of Hygiene and Tropical Medicine, Peru

## Abstract

**Objective:**

Growing evidence suggests high levels of comorbidity between hypertension and mental illness but there are few data from low- and middle-income countries. We examined the association between hypertension and depression and anxiety in South Africa.

**Methods:**

Data come from a nationally-representative survey of adults (n = 4351). The Composite International Diagnostic Interview was used to measure DSM-IV mental disorders during the previous 12-months. The relationships between self-reported hypertension and anxiety disorders, depressive disorders and comorbid anxiety-depression were assessed after adjustment for participant characteristics including experience of trauma and other chronic physical conditions.

**Results:**

Overall 16.7% reported a previous medical diagnosis of hypertension, and 8.1% and 4.9% were found to have a 12-month anxiety or depressive disorder, respectively. In adjusted analyses, hypertension diagnosis was associated with 12-month anxiety disorders [Odds ratio (OR) = 1.55, 95% Confidence interval (CI) = 1.10–2.18] but not 12-month depressive disorders or 12-month comorbid anxiety-depression. Hypertension in the absence of other chronic physical conditions was not associated with any of the 12-month mental health outcomes (p-values all <0.05), while being diagnosed with both hypertension and another chronic physical condition were associated with 12-month anxiety disorders (OR = 2.25, 95% CI = 1.46–3.45), but not 12-month depressive disorders or comorbid anxiety-depression.

**Conclusions:**

These are the first population-based estimates to demonstrate an association between hypertension and mental disorders in sub-Saharan Africa. Further investigation is needed into role of traumatic life events in the aetiology of hypertension as well as the temporality of the association between hypertension and mental disorders.

## Introduction

Chronic forms of morbidity, including mental disorders and hypertension, play a central role in shaping the burden of disease in the developing world. In South Africa there is a high prevalence of mental disorders, with an estimated 16% of adults living with an anxiety disorder and 10% with major depression [1]. Hypertension is a leading risk factor for mortality and morbidity worldwide, accounting for approximately 6% of global deaths [2]–[4]. The prevalence of hypertension in South Africa is over 20% [5].

A number of studies from Europe and North America have described an increased prevalence of chronic physical conditions among those with mental disorders [6], [7]. There have been mixed findings for an association between hypertension and anxiety disorders in developed countries, with conflicting results from studies using the same design, and using the same measurements. Some studies have shown a positive association between hypertension and anxiety in both crude and multivariate analyses [8]–[12]. Conversely, there are studies that show no crude or adjusted association between hypertension and anxiety [13]–[15]. Several studies have observed a positive crude association between hypertension and anxiety disorders that does not persist after adjustment [16]–[18]. Evidence is inconclusive and does not always include adjustment for relevant confounding variables, particularly traumatic life experiences.

Less evidence is available on the relationship between hypertension and depressive disorders. A handful of studies have suggested that depression may be more common among individuals with hypertension [9], [19]–[20] while a much larger body of evidence shows no association between hypertension and depression [12]–[15], [21]–[22]. Additional research found no crude or adjusted association between hypertension and depression [12]–[15], [18], [22]–[24].

Most of the literature investigates the relationship between hypertension and either depression or anxiety alone and few studies have examined comorbid depression and anxiety [12]. The relationship between comorbid anxiety-depression and chronic physical conditions was examined in the data from 17 countries that completed World Mental Health surveys [25]. Those with non-comorbid depressive disorder, non-comorbid anxiety disorder, and comorbid depression-anxiety were all more likely to have hypertension compared to persons with neither a depressive nor an anxiety disorder.

Limited evidence is available from developing countries. Furthermore, analyses need to consider important confounders such as trauma and other chronic conditions. Trauma has not previously been adjusted for, despite its potential to be associated with both hypertension and mental health disorders. Hypertension is often a risk factor for other chronic conditions, and therefore an observed association between hypertension and a mental health disorder may not persist after adjustment for other chronic conditions as the true association may be between more severe chronic conditions and the mental health disorder.

Despite the prevalence of mental disorders and chronic diseases such as hypertension in South Africa and other developing countries, few studies examine the relationship between these conditions in this setting. This paper investigates the associations between self-reported hypertension diagnosis and Diagnostic and Statistical Manual of Mental Disorders 4^th^ edition (*DSM-IV*) defined 12-month a) anxiety disorders b) depressive disorders and c) comorbid anxiety-depression. We hypothesized that hypertension and anxiety and depressive disorders will be associated even after adjusting for potential confounding variables including demographic and socioeconomic risk factors, substance use disorders, traumatic life events and other chronic physical conditions.

## Methods

This study was conducted according to the principles expressed in the Declaration of Helsinki. The study was approved by the Institutional Review Board of the University of Stellenbosch (Project Number “N06/07/134”). All patients provided written informed consent for the collection of samples and subsequent analysis.

The South African Stress and Health (SASH) study is a cross-sectional survey of mental health in the South African adult population. The study is part of the World Health Organization World Mental Health Survey Initiative [26]–[28]. Its rationale and design have been described in detail previously [26], [29].

SASH sampling and data collection were conducted between 2002 and 2004. The survey population included all resident South Africans 18 years and older who lived in households and hostels during the field period of the study. A three-stage probability sample design included a primary stage of stratification by enumerator area (EA, a unit of census administration), a second stage of sampling dwelling units within each EA and a final stage random sub-selection of a single adult respondent from each of the selected households.

The EA units provided the primary stage sampling units for the SASH sampling. The approximately 85,000 EAs were then assigned to one of 53 strata. These strata were defined based on the province, urban/rural status and the majority population group (African, Coloured, White or Indian). A random sample of 5 dwelling units was selected from each EA to be included in the study population and was subsequently contacted for interviews. Within each selected dwelling unit, a single adult respondent was selected to participate. Fieldworkers made up to three attempts to contact the selected participants. The survey had a high initial response rate of 87%.

Interviews were conducted in the homes of the selected participants by trained field interviewers. The interviewers were trained in psychiatric interviewing and conducted a structured diagnostic interview which was translated into seven of the national languages.

### Measures

#### Hypertension and other chronic conditions

Hypertension was assessed as self-reported lifetime diagnosis in the section on *Chronic conditions* in the questionnaire. Participants responded to the following question: “Did a doctor or other health professional ever tell you that you had any of the following illnesses: high blood pressure”. In addition to this binary measure, a four-level categorical variable combining hypertension and other chronic physical conditions was created. This variable was divided into none (no chronic physical condition), hypertension only, hypertension plus another chronic physical condition, and other chronic physical condition only. Chronic physical conditions other than hypertension included the following: arthritis or rheumatism, chronic back or neck problems, any other chronic pain, a stroke, a heart attack, heart disease, asthma, any other chronic lung disease like COPD (chronic obstructive pulmonary disease) or emphysema, diabetes or high blood sugar, an ulcer in your stomach or intestine, thyroid disease, a neurological problem, like multiple sclerosis, Parkinson's, or seizures, epilepsy or seizures, and cancer.

#### Mental Disorders

The World Mental Health pencil and paper (PAPI) version of the WHO Composite International Diagnostic Interview Version 3.0 (CIDI-3.0) was used to assess mental disorders according to the definitions and criteria of the DSM-IV [8]. Lifetime and 12-month *DSM-IV* diagnosis of the following anxiety disorders were included in this analysis: (i) panic disorder without agoraphobia, (ii) generalized anxiety disorder (GAD), (iii) social phobia, (iv) agoraphobia without panic disorder, and (v) posttraumatic stress disorder (PTSD). Lifetime and 12-month *DSM-IV* diagnosis of major and minor depression was also assessed. Substance use disorders were treated as a potential confounder. The variable for substance use disorders included lifetime *DSM-IV* diagnosis of alcohol abuse (with and without depression), alcohol dependence with abuse, drug abuse (with and without depression) and drug dependence with abuse. Earlier versions of the CIDI have been found to have good inter-rater and test-retest reliability [30] and in other WMH methodological studies there has been strong validity of CIDI diagnoses when compared to diagnoses based on blinded clinical reappraisal interviews [31].

#### Additional Variables

Socioeconomic status (SES) was measured using estimated household income, years of participant education, and participant employment. In addition, an asset index based on 17 items of individual and household wealth was used to capture variation of socioeconomic position in the developing-country setting [32]. These measures of asset ownership were used to construct an aggregate asset score, which was categorized into categories for 0–5, 6–12 and 13–17 assets.

In addition to reporting measures of SES (household income, education, employment status and asset index) individually, we standardized the raw income, education and asset index values, and summed them to create an aggregate measure of SES. This standardized measure was divided into quartiles for analysis corresponding to low, low-moderate, moderate-high and high SES [33].

Alcohol use was described based on the years when the participants drank the most and analysed a categorical variable of more than once a week, once a week to once a month, and less than once a month. Lifetime smokers were defined as those who had smoked more than 100 cigarettes in their lifetime, and current smokers were those who self-reported currently smoking. The measurement of traumatic life events was based on the Life Event schedule of the World Mental Health Survey and included experiences of crime, war, natural disasters, accidents and illness.

#### Analysis

Data were analysed using Stata Version 10.0 (Stata Corporation, College Station, USA). All analyses reported accounted for the complex survey design based on person-level weights that incorporated sample selection, non-response and post-stratification factors. All statistical tests were two-sided at α = 0.05.

Descriptive statistics were generated with continuous variables reporting means and categorical data reporting proportions. The prevalence and proportions of the demographic and socioeconomic variables, as well as other variables (alcohol use, smoking, chronic physical conditions and traumatic life events), were examined among the total sample, and stratified by hypertension, anxiety disorders (lifetime and 12-month), depressive disorders (lifetime and 12-month), and comorbid anxiety-depression (lifetime and 12-month). The odds ratios (OR) and 95% confidence intervals (CI) of anxiety disorders, depressive disorders, and comorbid anxiety-depression by demographics, socioeconomic and other variables were generated with those with no mental disorder (no anxiety or depression) as the reference group.

The prevalence of hypertension and other chronic physical conditions in those with mental disorders (anxiety, depression and comorbid anxiety-depression), or the physical-mental comorbidity prevalences, were calculated for both lifetime and 12-month mental disorders. For each crude association, Pearson's chi-squared test used to compare proportions was calculated with the reference group being those without anxiety or depression. In addition, age adjusted odds ratios, with the reference group being those without anxiety or depression, with 95% confidence intervals and Pearson's chi-squared test for comparison of proportions were calculated for the physical-mental comorbidities.

We developed a series of multiple logistic regression models to assess the independent association between, 1) hypertension and anxiety disorders, 2) hypertension and depressive disorders, and 3) hypertension and comorbid anxiety-depression. Models for both hypertension as a binary variable (yes/no) and categorical variable including other chronic physical conditions (no chronic physical condition, hypertension only, hypertension and another chronic physical condition, and another chronic physical condition) were built. The models included adjustment for demographics, an aggregate measure of SES, lifetime smoking and alcohol use, substance use disorders and traumatic life events.

## Results

The demographic characteristics and socioeconomic characteristics of the study sample are presented in Table 1. The mean age was 37 years and half of the sample was married (50%). 76% of the sample was Black, 10% Coloured, 10% White and 3% Indian/Asian. Less than a third of the sample was employed (31%) and 74% had completed at least some high school. Of the total sample, 8% had a 12-month anxiety disorder, 5% a 12-month depressive disorder and 1% had 12-month comorbid anxiety-depression (Table 2).

**Table 1:** Description of sample, stratified by hypertension diagnosis.

	Total	Hypertension diagnosis	No hypertension diagnosis	p-value
	%	%	%	
N (%)	4351	767 (16.7)	3584 (83.3)	
**Demographic Characteristics**				
Mean Age	37.0	50.3	34.3	-
Age categories: 18–29	39.1	9.0	45.1	<0.001
30–39	22.1	13.5	23.8	
40–49	18.1	24.2	16.9	
50+	20.7	53.3	14.2	
Sex: Male	46.3	28.0	50.0	<0.001
Female	53.7	72.0	50.0	
Race: Black	76.2	76.1	76.3	0.271
Coloured	10.4	11.7	10.2	
White	10.0	10.2	9.9	
Indian/Asian	3.4	2.0	3.6	
Currently married	50.1	54.0	47.1	<0.001
Location: Rural	38.4	41.6	37.7	0.074
Urban	61.6	58.5	62.3	
**Socioeconomic status**				
Education: None	6.8	12.7	5.6	<0.001
Grade 1–7	19.1	33.9	16.2	
Grade 8–11	35.4	32.9	35.9	
Completed high school	23.5	11.4	25.9	
Post-high school education	15.3	9.2	16.5	
Employed	31.0	26.0	32.0	0.020
Household income (mean)	59403.9			
R0	13.7	13.3	13.7	0.244
R1–5000	29.5	32.9	28.9	
R5001–25000	15.4	16.7	15.1	
R25000–100000	19.6	17.4	20.1	
R100001+	21.8	19.7	22.3	
Assets owned by household: 0–5	39.3	38.3	39.5	
6–12	37.4	41.0	36.7	
13–17	23.3	20.7	23.8	0.177
SES Quartile: 0	22.5	36.0	19.8	<0.001
1	24.5	22.1	24.9	
2	25.0	20.8	25.9	
3	28.0	21.0	29.4	
**Other**				
Alcohol: Lifetime – None	77.8	79.1	77.5	0.157
Rare	5.8	7.0	5.5	
Moderate	7.5	5.7	7.9	
Heavy	8.9	8.2	9.1	
Alcohol: Current – None	65.7	71.8	64.5	0.053
Rare	10.2	8.7	10.5	
Moderate	16.8	13.5	17.4	
Heavy	7.3	6.0	7.6	
Smoking				
Lifetime smoker	30.0	26.1	30.8	0.033
Current smoker	23.8	15.9	25.4	<0.001
Chronic physical conditions	42.6	78.5	35.4	<0.001
Vascular	11.2	40.2	5.4	<0.001
Other	39.4	69.9	33.3	<0.001
Traumatic life events				
None	26.6	17.3	28.5	<0.001
1–2	49.9	52.5	49.4	
3–4	10.8	11.9	10.6	
5 or more	12.7	18.3	11.5	

**Table 2:** Description of sample by 12-month *DSM-IV* Anxiety & Major Depression.

	No depression or anxiety	Anxiety	OR (95% CI)	Major Depression	OR (95% CI)	Comorbid anxiety-depression	OR (95% CI)
	%	%		%		%	
Prevalence	87.8	8.1		4.9		1.4	
Mean Age	36.8	38.4		37.6		39.5	
Age categories:18–29	39.8	33.3	1.0	32.2	1.0	22.9	1.0
30–39	21.9	23.2	1.3 (1.0–1.7)	24.4	1.4 (0.9–2.1)	30.8	2.4 (1.0–6.0)
40–49	17.6	21.2	1.4 (1.0–2.1)	23.3	1.6 (1.1–2.5)	20.9	2.1 (1.0–4.2)
50+	20.7	22.3	1.3 (0.8–2.0)	20.2	1.2 (0.8–1.8)	25.4	2.1(1.0–4.5)
Sex: Male	48.4	30.1	1.0	29.2	1.0	11.3	1.0
Female	51.7	69.9	2.2 (1.6–2.9)	70.8	2.3 (1.6–3.2)	88.7	7.4 (3.4–16.0)
Race: Black	76.2	79.9	1.0	71.8	1.0	79.8	1.0
Coloured	10.1	11.5	1.1 (0.7–1.7)	13.4	1.4 (0.9–2.1)	9.7	0.9 (0.3–2.4)
White	10.4	6.5	0.6 (0.2–1.6)	7.6	0.8 (0.3–2.1)	7.7	0.7 (0.1–5.9)
Indian/Asian	3.2	2.1	0.6 (0.3–1.3)	7.2	2.4 (1.1–5.0)	2.8	0.8 (0.2–3.1)
Currently married	50.1	48.6	0.9 (0.7–1.2)	53.1	1.1 (0.9–1.5)	50.9	1.0 (0.6–1.7)
Location: Urban	61.2	66.1	1.2 (0.9–1.6)	65.2	1.2 (0.9–1.7)	76.2	2.0 (1.1–2.6)
Hypertension diagnosis	15.7	26.9	2.0 (1.4–2.8)	21.2	1.4 (1.0–2.0)	31.6	2.4 (1.2–5.1)
Lifetime smoker	29.0	34.6	1.3 (1.0–1.6)	38.9	1.6 (1.1–2.2)	27.0	0.9 (0.5–1.7)
Current smoker	23.2	24.6	1.1 (0.9–1.4)	31.1	1.5 (1.0–2.2)	19.0	0.8 (0.4–1.6)
Other chronic physical condition	40.3	59.8	2.2 (1.7–2.8)	59.8	2.2 (1.6–3.1)	67.8	3.1 (1.6–6.2)
Vascular	10.2	20.0	2.2 (1.5–3.3)	16.3	1.7 (1.1–2.6)	21.8	2.5 (1.0–5.8)
Other	37.1	57.8	2.3 (1.8–3.0)	56.2	2.2 (1.5–3.1)	64.6	3.1 (1.6–6.1)
Traumatic life events: None	28.3	16.8	1.0	10.0	1.0	10.2	1.0
1–2	50.2	45.0	1.5 (1.0–2.2)	51.5	2.9 (1.7–4.9)	40.6	2.3 (0.9–5.6)
3–4	10.4	13.0	2.1 (1.3–3.5)	15.7	4.2 (2.4–7.6)	19.9	5.3 (1.9–14.7)
5 or more	11.1	25.2	3.8 (2.6–5.7)	22.8	5.8 (3.6–9.4)	29.4	7.4 (2.7–20.3)

Overall, 17% of participants reported being told that they had hypertension. More than forty percent of the sample (43%) had at least one chronic physical condition, and 79% of those with hypertension had at least one chronic condition (Table 1). Strong crude associations were found between hypertension diagnosis and age, sex, marriage, education, employment status, smoking (current and lifetime), chronic physical conditions, and traumatic life events (p-values all <0.001). Women were 2.6 times more likely to report a lifetime diagnosis of hypertension compared to men (p<0.001). People with another chronic condition were 6.7 times more likely to report a lifetime diagnosis of hypertension compared to those without a hypertension diagnosis (p-<0.001). Among measures of socioeconomic status, those with a hypertension diagnosis were less educated and more likely to be unemployed. The aggregate measure of SES was strongly associated with hypertension; those with a hypertension diagnosis had a lower SES than those without a hypertension diagnosis (Table 1).

Table 2 presents some of the demographic and other characteristics of those with and without 12-month anxiety and depressive disorders. Females were more than twice as likely to have 12-month anxiety or depressive disorders (OR = 2.2, 95% CI = 1.6–2.9; OR = 2.3, 95% CI = 1.6–3.2), and more than seven times more likely to have comorbid anxiety-depression compared to men (OR = 7.4, 95% CI = 3.4–16.0). Those with mental disorders also reported an increased prevalence of chronic conditions other than hypertension with significantly more reporting being diagnosed as hypertensive. Those with a 12-month anxiety disorder were twice as likely to report a lifetime diagnosis of hypertension and twice as likely to report another chronic condition (OR = 2.0, 95% CI = 1.4–2.8; OR = 2.2, 95% CI = 1.7–2.8). Traumatic life events were also highly associated with all 12-month mental disorders. Those with a 12-month depressive disorder were 2.9 times more likely to report 1 or 2 traumatic life events, 4.2 times more likely to report 3 or 4 traumatic life events and 5.8 times more likely to report 5 or more traumatic life events compared to those without a 12-month depressive disorder (Table 2).

There was variability in the association between a recent diagnosis of hypertension and specific mental disorders during the previous 12 months (Table 3). Hypertension was more commonly reported in participants with agoraphobia, generalized anxiety disorder and panic disorder, but was not increased in individuals with PTSD or social phobia. Major depression was associated with an increased prevalence of hypertension. Overall, those with a 12-month mental disorder were 1.68 times more likely to report being diagnosed as hypertensive compared to those without a 12-month mental disorder.

**Table 3:** Prevalence and relative odds of 12-month mental disorders by past hypertension diagnosis.

	Total	Hypertension diagnosis	No hypertension diagnosis	p-value	OR (95% CI)
	% (n)	%			
Any anxiety disorder	8.23 (375)	26.92	15.8	<0.001	1.97 (1.41–2.75)
Agoraphobia	5.13 (232)	22.7	16.4	0.042	1.50 (1.01–2.22)
Generalized anxiety disorder	1.91 (90)	41.0	16.2	<0.001	3.59 (2.13–6.05)
Panic disorder	0.79 (37)	39.0	16.5	0.002	3.23 (1.51–6.93)
PTSD	0.58 (27)	25.6	16.6	0.232	1.72 (0.69–4.31)
Social phobia	1.88 (87)	19.4	16.6	0.475	1.21 (0.71–2.05)
Any depressive disorder	5.4 (249)	21.2	16.4	0.060	1.37 (0.99–1.90)
Major depressive disorder	4.8 (223)	23.0	16.4	0.020	1.52 (1.07–2.17)
Minor depressive disorder	0.6 (26)	6.7	16.8	0.076	0.36 (0.11–1.18)
Comorbid anxiety-depression	1.4 (67)	31.6	16.5	0.019	2.34 (1.14–4.83)
Any anxiety or depressive disorder	12.3 (557)	23.9	15.8	<0.001	1.68 (1.31–2.16)

Table 4 presents the association between hypertension and mental health disorders in models that do and do not adjust for other chronic conditions as well as adjusting for a range of other variables. Without adjusting for other chronic conditions, self-reported hypertension is associated with 12-month anxiety disorders (OR = 1.55) but not with 12-month depressive disorders (p-value) or 12-month comorbid anxiety-depression (p-value) (Table 4). When other chronic conditions are included in the final model, there is no association between hypertension (in the absence of another chronic condition) are mental health disorders. However, hypertension and other chronic condition are associated with 12-month anxiety disorders (OR = 2.25). Furthermore, other chronic conditions are associated with 12-month anxiety (OR = 1.74), depressive (OR = 1.56), and comorbid anxiety-depressive disorder (OR = 2.35) (Table 4).

**Table 4:** Multivariate models examinating the association between 12-month mental disorders and hypertension*.

Model	Hypertension variable(s)	12-month anxiety disorders	12-month depressive disorders	12-month comorbid anxiety-depression
		OR (95% CI)	OR (95% CI)	OR (95% CI)
Model A – Hypertension as a binary variable	Hypertension diagnosis	1.55 (1.10–2.18)	1.01 (0.68–1.50)	1.38 (0.60–3.18)
Model B – Hypertension as a categorical variable including other chronic physical conditions	Hypertension diagnosis only	1.58 (0.74–3.38)	0.81 (0.35–1.87)	2.74 (0.81–9.22)
	Hypertension and another chronic physical condition	2.25 (1.46–3.45)	1.44 (0.91–2.29)	2.14 (0.82–5.63)
	Another chronic physical condition	1.74 (1.28–2.37)	1.56 (1.07–2.26)	2.35 (1.10–5.01)

* Models A and B are both adjusted for demographic variables (age, sex, race marriage, location), SES, lifetime smoking and alcohol use, substance use disorders and traumatic life events.

Table 5 presents the multivariate models examining the association between 12-month mental health disorders and participant demographic, socioeconomic and health characteristics. After adjustment, females were 3 times more likely to have a 12-month anxiety disorder or depressive disorder, and more than 12 times more likely to have 12-month comorbid anxiety-depressive disorder compared to men. Furthermore, independent of hypertension status, those with 5 or more traumatic life events were more likely to have a 12-month anxiety disorder, depressive disorder, and co-morbid anxiety-depressive disorder compared to those without a traumatic life event (p-values all <0.05).

**Table 5:** Summary of multivariate models examining the association between hypertension and 12-month mental health outcomes*.

	Anxiety		Depression		Comorbid anxiety-depression	
	OR	95% CI	OR	95% CI	OR	95% CI
Hypertension variable						
None	1.0		1.0		1.0	
Hypertension diagnosis only	1.58	0.74–3.38	0.81	0.35–1.87	2.74	0.81–9.22
Hypertension diagnosis and chronic	2.25	1.46–3.45	1.44	0.91–2.29	2.14	0.82–5.63
Chronic only	1.74	1.28–2.37	1.56	1.07–2.26	2.35	1.10–5.01
Age: 18–29	1.0		1.0		1.0	
30–39	1.09	0.80–1.47	1.17	0.74–1.85	1.95	0.82–4.62
40–49	1.03	0.68–1.56	1.27	0.78–2.07	1.30	0.68–2.47
50+	0.94	0.56–1.56	0.97	0.62–1.52	1.76	0.83–3.70
Sex: Male	1.0		1.0		1.0	
Female	3.24	2.25–4.67	3.47	2.33–5.15	12.50	4.59–34.04
Race: Black	1.0		1.0		1.0	
Coloured	0.74	0.44–1.24	1.00	0.65–1.54	0.49	0.18–1.32
White	0.43	0.17–1.09	0.57	0.27–1.24	0.41	0.06–2.68
Indian/Asian	0.48	0.21–1.07	1.96	0.95–4.05	0.52	0.13–2.15
Currently married	0.87	0.66–1.13	0.98	0.72–1.33	0.86	0.51–1.44
Location: Rural	1.0		1.0		1.0	
Urban	1.36	1.00–1.85	1.09	0.75–1.58	2.08	1.18–3.65
SES Quartile – 0	1.0		1.0		1.0	
1	0.95	0.64–1.43	1.19	0.77–1.81	1.35	0.71–2.59
2	0.85	0.56–1.28	0.91	0.58–1.41	1.24	0.54–2.85
3	1.01	0.63–1.63	1.04	0.61–1.78	1.28	0.43–3.78
Alcohol: Lifetime – None	1.0		1.0		1.0	
Rare	1.29	0.65–2.54	1.96	1.00–3.84	2.75	0.53–14.40
Moderate	1.25	0.67–2.32	1.91	1.11–3.29	2.91	0.89–9.55
Heavy	1.47	0.81–2.67	1.14	0.61–2.11	3.23	1.28–8.17
Lifetime smoker	1.57	1.20–2.06	2.03	1.34–3.08	1.28	0.46–3.52
Substance use disorder	2.32	1.32–4.09	1.44	0.83–2.52	1.73	0.67–4.47
Traumatic life events – None	1.0		1.0		1.0	
1–2	1.15	0.77–1.70	2.44	1.44–4.14	1.52	0.61–3.75
3–4	1.44	0.88–2.37	3.36	1.91–5.91	3.18	1.16–8.76
5 or more	2.62	1.70–4.03	4.27	2.49–7.32	4.49	1.59–12.65

* All models are adjusted for demographic variables (age, sex, race marriage, location), SES, lifetime smoking and alcohol use, substance use disorders and traumatic life events.

## Discussion

This study suggests that self-reported diagnosis of hypertension is more common among South Africans with 12-month anxiety disorders, depressive disorders and comorbid anxiety-depression compared to those without a mental disorder. However, hypertension diagnosis without another chronic physical condition (hypertension only) was not associated with any of the mental health outcomes (anxiety, depression, and comorbid anxiety-depression) in multivariate models. Hypertension diagnosis and another chronic condition were consistently associated with anxiety disorders, depressive disorders and comorbid anxiety-depression after adjustment for various confounding variables. Therefore, adjusting for other chronic conditions explains the observed crude associations between mental health disorders and hypertension.

This analysis makes significant advances on previous studies of this association. This is the first population-based study from sub-Saharan Africa to document an association between anxiety and depressive disorders and hypertension. Our analysis included adjustment for traumatic life events which has previously never been done; given the strong associations between life events and both hypertension and common mental disorders, accounting for this covariation is an important consideration. In addition, few other studies of the association between hypertension and mental disorders have included other chronic conditions as a potential confounder.

Our evidence for an association between hypertension and anxiety disorders after adjusting for demographics, SES, lifetime smoking and alcohol behaviour, substance use disorders and traumatic life events is similar to the majority of studies in the literature [8], [12]. The observed odds ratio of 1.6 may be smaller than those found in previous studies as we adjusted for a larger number of potential cofounders. Our principle confounding factor appeared to be traumatic life events, a variable that has previously never been considered in this association. The findings add to the previous evidence of an association between hypertension and anxiety disorders as well as providing evidence that the association exists in a developing country context.

Major depressive disorder demonstrated a positive crude association with hypertension diagnosis that did not persist in multivariate analysis when adjustment was made for demographics and traumatic life events. These results are similar to the majority of studies in the literature which suggests no association, or a crude association that does not persist in multivariate analysis between hypertension and depressive disorders.

In our study, the association with hypertension and another chronic physical condition was attenuated after adjustment for demographics and traumatic life events However, failure to show an adjusted association between hypertension and comorbid anxiety-depression may be the result of a lack of statistical power as only 67 people had comorbid anxiety-depression.

The study sample is nationally representative which gives it strong generalisability to the country and meaningful insight into the burden of hypertension and mental health in the country. Furthermore, with the exception of one study from Zimbabwe [35], this is the first large scale study of the association between hypertension and mental health in an African and developing country context.

There are several notable limitations to these results. The cross-sectional design limits the ability to ascertain temporality between hypertension diagnosis and mental health outcomes. The use of self-reported lifetime diagnosis of hypertension as the hypertension measure is a limitation of the study. Self-reporting may introduce measurement bias, where those who have a mental health disorder are more likely to recall a diagnosis of hypertension thus inflating the true association between hypertension and mental health disorders. Furthermore, self-reported hypertension is generally underreported [36]. Previous research suggests that measured blood pressure is modestly associated with self-reported hypertension status. However, reassurance is obtained from previous data which indicate that self-reported hypertension is moderately associated with objective data on hypertensive status [37]–[38]. The prevalence of self-reported hypertension from this data was 17% which is less than the 21% reported by the 1998 South African Demographic and Health Survey which measured hypertension at the time of administering the questionnaire [4].

Mental health was assessed using the CIDI 3.0, an instrument designed in the context of developing countries [39]. A significant body of literature is available on the cross-cultural challenges in measuring mental health. The literature highlights two primary issues; one on the linguistic issues regarding comprehension and understanding of mental health constructs and one on the socio-cultural nature of mental health and how the symptoms may manifest differently in different societies [40]–[41]. As an example, it has been recognized that depression for black Africans may present with different linguistic phrases and symptoms may both occur in different places and in different ways to those of Western culture [40]. South Africa is a heterogeneous society, with significant diversity in cultures. The CIDI 3.0 has not been validated for South Africa, with research on the concordance of the CIDI compared to standardized clinical interviews for *DSM-IV* diagnosis (SCID) done only in France, Italy, Spain and the United States. The results show the agreement to be good, with CIDI 12-month prevalences generally conservative relative to SCID [31]. There is potential for this measurement to introduce bias to the results, both through random and systematic misclassification. Random misclassification may have happened if the misclassification of mental disorders occurred to the same degree among those with and without hypertension diagnosis.

A strength of the dataset is that information is available on a number of potential confounders that have not been accounted for in previous studies of this association We also had information on a large number of chronic physical conditions, both conditions in the past 12-months and lifetime diagnoses from health care professionals. Adjustment for other chronic physical conditions proved highly important, demonstrating that hypertension on its own has no association with anxiety, depression or comorbid anxiety-depression in crude or adjusted analyses. We were able to adjust for demographics and socioeconomics, as well as lifestyle risk factors (smoking and alcohol use) and substance use disorders.

There is a high prevalence of hypertension and mental health disorders in South Africa. The comorbidity observed in developing countries between chronic physical conditions and mental disorders is also present in the South African context. Multivariate analysis adjusting for other chronic physical conditions and traumatic life events show a smaller than previously presented association between hypertension and mental health disorders.
